RETRACTED

# Clinical Effect of Microneedle Injection Combined with Blood Transfusion in the Treatment of Severe Anemia Complicated with Vitiligo under Regenerative Medical Technology

**DOI:** 10.1155/2022/7117627

**Published:** 2022-07-29

**Authors:** Tao He, Li Gong

**Affiliations:** ^1^Blood Transfusion Department, Beidahuang Group General Hospital, Harbin, 150088 Heilongjiang, China; ^2^Department of Dermatology, The First Hospital of Heilongjiang Harbin, Harbin, 150010 Heilongjiang, China

## Abstract

To explore the clinical efficacy of microneedle injection combined with blood transfusion in the treatment of severe anemia complicated with vitiligo based on regenerative medical technology and provide the theoretical basis for the adoption of microneedle technology, 60 patients with severe anemia complicated with vitiligo were selected as research objects. With 15 patients in each group, they were randomly assigned to the control group (calcipotriol ointment external application), observation group A (external application of moist exposed burn ointment (MEBO), observation group B (external application of MEBO combined with blood transfusion), and observation group C (microneedle injection of MEBO combined with blood transfusion). Blood indexes and plaque recovery of patients in different periods were detected. The total protein (TP) content in group C (62.3 ± 3.3 g/L and 64.3 ± 2.88 g/L) was remarkably higher than that in the control group (51.3 ± 3.17 g/L and 52.4 ± 3.17 g/L) and group A (52.6 ± 2.91 g/L and 51.8 ± 2.98 g/L)) at the 5th and 7th weeks after the treatment (*P* < 0.05). The albumin (ALB) content in group C (42.9 ± 3.28 g/L and 45.3 ± 3.1 g/L) was signally higher than that in the control group (41.8 ± 3.44 g/L and 41.9 ± 3.23 g/L) and group A (41.3 ± 2.91 g/L and 42.1 ± 3.02 g/L) at the 5th and 7th weeks after the treatment, and the content was markedly higher than that in group B at 5th week (*P* < 0.05). The wound healing rates of group C at the 3rd, 5th, and 7th weeks after the treatment (38.44%, 56.6%, and 90.23%) were greatly higher than those of the control group, group A, and group B (*P* < 0.05). Besides, the wound healing rate of group B was higher than that of the control group and group A (40.3% and 75.8%) at the 5th and 7th weeks after the treatment (*P* < 0.05). To sum up, based on regenerative medical technology, microneedle injection (microneedling is a derma roller process that pricks the skin with minuscule needles. The goal of the treatment is to develop new collagen and skin tissue, resulting in skin that is smoother, firmer, and more toned) combined with blood transfusion had a good therapeutic effect on patients with severe anemia complicated with vitiligo, which could manifestly improve the blood indexes and skin plaques of patients, with a good clinical adoption effect.

RETRACTED

## 1. Introduction

Severe anemia refers that when the haemoglobin concentration is too low, the patient has some serious ischemia or anoxic symptoms, such as dizziness, lack of power, palpitation, bosom frowsty, weakness, fatigue skin that is pale or yellowish, heartbeat irregularities, breathing problems, light-headedness or dizziness chest discomfort, hands, and feet are freezing, and headaches. Anemia might be so subtle at first that it goes unnoticed. However, as anemia worsens, symptoms worsen, as does breathing difficulty. Mild anemia, moderate anemia, and severe anemia refer to haemoglobin concentrations below normal but greater than 90 g/L, 60 g/L, and 89 g/L and less than 60 g/L, respectively [1, 2]. Some factors can cause severe anemia, such as decreased erythropoiesis, increased damage to erythrocytes, and blood loss. Clinical manifestations are often the pallor of skin and mucosa, tachypnoea, aggravation of fatigue, muscle weakness, etc. Moreover, there are even dyspnoea, nausea, abdominal pain, abdominal distension, chest tightness, and shortness of breath in a calm state [3]. If severe anemia occurs, patients need to go to the hospital for treatment in time. Patients need to stay in bed as much as possible and receive oxygen inhalation and blood transfusion treatment. Besides, when their conditions become stable, they need to receive the targeted treatment, such as iron supplementation and folic acid vitamin supplementation [4, 5]. Vitiligo is a common chronic immune skin disease mainly characterized by white plaques (Candida oral lesions occur as white plaques or patches, frequently with a milk curd appearance, that wipes away with pressure, leaving a red, sometimes hemorrhagic surface. The buccal mucosa, tongue, and palate are the most typically affected areas) at the exposed skin sites. It is mainly manifested as decreased skin color and white plaques on the skin, which can gradually expand or even appear as multiple white plaques. In severe cases, the skin of the whole body can become white [6, 7].

The white plaques on the body's sides are banded distribution, and patients' appearance and mentality are affected. The pathophysiology of vitiligo is still a mystery. It has a connection with immunological factors, genetic factors, and neurological issues in general. Vitiligo has been linked to autoimmune and endocrine problems in a few cases [8, 9]. The disease is a refractory disease with a protracted and difficult treatment cycle, whereas patients with a brief disease phase have an optimal therapeutic outcome. Through active treatment, the skin appearance can be effectively improved, and even the skin color can be restored. However, there is a risk of relapse [10]. Anemia can cause the relapse of vitiligo. At present, although there is not a clear conclusion for the pathogenesis, vitiligo is associated with low immunity in the human body to some extent. The incidence of vitiligo increases notably when patients are in a state of disease or poor physical condition [11, 12]. Anemia can lead to low immunity and slow metabolism, and vitiligo, as a disease that is difficult to cure, has a high possibility of relapse [13, 14]. Moreover, the history of vitiligo and anemia increases the risk of vitiligo relapse. Many patients with vitiligo are accompanied by anemia. Anemia and hematopoietic dysfunction will cause immune dysfunction that results in the decline of patients' resistance and immunity [15, 16].

RETRACTED

Meanwhile, anemia can cause inappetence, so patients receive various infectious diseases, which is not conducive to the rehabilitation of vitiligo [17]. Microneedle therapy is stimulating the skin with several needles on the microneedle roller to make some tiny tubes within a short time so that the active substance can effectively penetrate the skin to achieve a good therapeutic effect [18]. This treatment has the advantages of a short recovery period, rapid healing, no scars, and small side effects, and it is widely applied. It is of great value in the treatment of skin diseases [19]. However, there are many strict indications of the use of microneedles. Patients with healthy skin barriers can benefit from needle rolling. The depth and strength of microneedles should be considered for patients with inadequate skin barriers. The fundamental goal of regenerative medical technology is to regenerate the surviving living tissue cells on the wound into new tissue cells in situ, as well as regenerate new tissue and skin after the culture [20]. The adoption of regenerative medical technology plays a key role in the in situ regeneration of skin organs and the promotion of the healing of injured skin. Nevertheless, there are few investigations on the adoption value of regenerative medicine techniques (these treatments could include biochemical approaches to stimulate tissue regeneration directly at the site of injury or transplantation techniques using differentiated cells or stem cells, either alone or as part of a bioartificial tissue. Seeding cells onto natural or biomimetic scaffolds produce bioartificial tissues) in the treatment of anemia complicated with vitiligo. Hence, under the regenerative medical technology combined with microneedle introduction, it was used in the treatment of severe anemia complicated with vitiligo to analyse its curative effect and clinical adoption value.

RETRACTED

The rest of the paper is organized as Section 2 gives material and methods, Section 3 gives us results, Section 4 gives us discussion, and the conclusion is given in Section 5.

## 2. Materials and Methods

In this section, we will discuss research objects and grouping, the introduction of microneedles under regenerative medical technology, treatment of patients, observation indexes, and statistical methods in detail.

### 2.1. Research Objects and Grouping

60 patients with severe anemia complicated with vitiligo who were treated in The First Hospital of Heilongjiang Harbin from January 2017 to November 2020 were selected as the research objects. There were 28 male patients and 32 female patients whose ages ranged from 20 to 55 years old, with an average age of 25.38 ± 6.54 years old. They were randomly divided into the control group (external application of calcipotriol ointment—calcipotriene is a vitamin D derivative. It works by reducing the rate at which skin cells proliferate), the observation group A treated with external application of moist exposed burn ointment (MEBO), the observation group B (external application of MEBO combined with blood transfusion), and the observation group C (microneedle injection of MEBO combined with blood transfusion), with 15 patients in each group. This experiment was approved by the *Medical Ethics Committee of* The First Hospital in Heilongjiang Harbin. Patients and their families understood the content and methods and agreed to sign the informed consent.

The inclusion criteria were as follows:

1. Patients with vitiligo plaques in multiple exposed parts, including the face and neck, trunk, and limbs
2. Patients with no history of vitiligo and anemia and no oral drug therapy, topical drug application, or surgical treatment
3. Patients who agreed to microneedle therapy
4. Patients with skin pigment depigment plaques and the affected part in milky white or different shapes

The exclusion criteria were as follows:

1. Patients with other systemic diseases or serious infectious diseases
2. Patients with incomplete clinical data and information
3. Patients who recently were treated with other medications

### 2.2. Introduction of Microneedles under Regenerative Medical Technology

Based on the medical theory of skin regeneration in situ, the MEBO (Shantou MEBO Pharmaceutical Co., Ltd.) that helped to promote the proliferation and differentiation of epidermal stem cells was used for the treatment of patients with severe anemia complicated with vitiligo. Microneedles were used to stimulate the skin, and numerous tiny tunnels were produced on the skin to allow the active substances to penetrate. The rolling of the microneedle could stimulate the dermis of the skin, causing collagen and fibroblasts to proliferate [21, 22]. The patient's healthy skin (abdomen and buttocks) was firstly punctured with hollow microneedles. Then, the skin in the leucoplakia area was punctured with microneedles to achieve the transplantation of vitiligo melanocytes. The drug was introduced into the skin using microneedle technology to cause epidermal stem cells in situ to hyperplasia, differentiate into melanocytes, and repair the damaged melanocytes, effectively improving the microcirculation of the injured part of the patient, repairing the leucoplakia, and potentially helping to treat vitiligo.  Figure 1 shows the principle of the drug introduced by the microneedles.

RETRACTED

### 2.3. Treatment of Patients

In the control group, 75% medical alcohol was used to routinely disinfect the white spot and its surrounding skin. After the disinfection, the calcipotriol ointment (Shanghai Chemvon Biochemical Technology Co., Ltd.) was applied to the white spot once a day, for one month for a course of treatment, for three courses of continuous treatment. Blood analysis was performed in groups A, B, and C, including haemoglobin, blood glucose, fasting blood glucose, white blood cells, and neutrophils. The symptoms and risks of anemia, as well as the aim and precautions of blood transfusion, were thoroughly discussed with patients and their families. Vital signs of patients were monitored in real time before and after transfusion. 200 mL blood was transfused, with 15 mL/h for the first 15 min, and it was gradually increased to 30 mL/h until the transfusion was completed.

In group A, the MEBO was applied to the white plaques for external use, and the application scope, dosage, and application time were consistent with those of the control group. In group B, based on blood transfusion and transfusion nursing, MEBO (Shantou MEBO Pharmaceutical Co., Ltd.) was applied to the white plaques, and the scope, dosage, and time of application were consistent with those of the control group.

In group C, based on transfusion therapy and transfusion nursing, the patients were treated with MEBO combined with microneedle based on regenerative medical technology. The skin lesions and white plaques of patients were disinfected. After the disinfected parts were dry, the skin was tightened. 2.0 mm microneedle (Guangzhou YOUTH Science and Technology Co., Ltd.) was used to roll back and forth at the lesion sites, and the rolling range of the microneedle was greater than 2 cm^2^ of the lesion site area. Each skin lesion site was rolled for about 5 minutes until the skin became red, and there was slight oozing of blood. Microneedle rolling was stopped, and bleeding spots were removed with a sterile cotton ball. A small amount of MEBO was dipped by a cotton swab, and it was evenly applied to the skin of the rolling area, and the thickness of the application was about 2 mm. The area where the drug was applied was covered with sterile gauze. Skin microneedles were punched once a week, and the drug was applied once a day, and it was covered with gauze after the application.

RETRACTED

### 2.4. Observation Indexes

After treatment, blood indexes of patients in the four groups were measured at the 1st, 3rd, 5th, and 7th weeks, including white blood cells, the absolute value of neutrophil, the total number of lymphocytes, albumin (ALB), globulin (GLB), and total protein (TP). The efficacy of vitiligo treatment was assessed after 3 months.  Table 1 shows the methods.

According to the above efficacy evaluation criteria, the recovery effects of all patients were evaluated, and Equation (1) shows how the treatment effective rate (*R*) was calculated.

(1) $$\begin{array}{c} R=\left[\frac{\left(A+B+C\right)n}{N}\right]\times 100\%. \end{array}$$

In Equation (1), *n* represents the number of cases, and *N* represented the total number of cases. *A*, *B*, and *C* represented the recovery, clinical marked effect, and improvement, respectively. Equation (2) shows how the wound healing rate of patients was calculated.

(2) $$\begin{array}{c} \text{Healing rate}=\left(\frac{S_{0}-S_{1}}{S_{0}}\right)\times 100\%. \end{array}$$

In Equation (2), *S*_0_ expressed the area of white plaques before treatment and *S*_1_ expressed the area of white plaques after treatment.

### 2.5. Statistical Methods

SPSS 22.0 was employed for data statistics and analysis. Mean ± standard deviation ($\bar{x}\pm s$) was how measurement data were expressed, and percentage (%) was how count data were expressed. Analysis of variance was used for the pairwise comparison. The difference was statistically significant with *P* < 0.05.

## 3. Results

In this section, we will discuss the blood indexes of patients before treatment, microscopic images of the skin of patients with vitiligo, changes in blood biochemical indexes of patients, the skin improvement of patients, evaluation of therapeutic effects, and comparison of wound healing rate of patients in detail.

### 3.1. Blood Indexes of Patients before Treatment

Figure 2(a) shows the comparison of absolute values of white blood cells, neutrophils (neutrophils are the most common leukocytes in circulation and have long been recognized as the innate immune system's first line of defense. After recognizing pathogens, they use phagocytosis and intracellular degradation, as well as the release of granules and the development of neutrophil extracellular traps, to collect and eliminate invading bacteria), and the total number of lymphocytes in the control group, group A, group B, and group C before treatment.  Figure 2(b) shows the comparison of ALB content, and Figure 2(c) shows that of GLB content. There were insignificant differences in blood indexes of patients with severe anemia in the four groups before transfusion (*P* > 0.05).

RETRACTED

### 3.2. Microscopic Images of the Skin of Patients with Vitiligo

Figure 3 shows the microscopic images of the skin of patients with vitiligo. Dermis belonged to the irregular dense connective tissue, which was composed of fibers, matrix, and cell components, mainly the fiber components. The collagen and elastic fibers were woven together, as were the rich thick collagen fibers, to produce a dense lamellar structure. Fibers contained a limited quantity of matrix and cell components. In Figure 3, the microscopic images of the skin of patients with vitiligo showed that melanin cells and melanin particles were decreased or even disappeared. There were epidermal hyperkeratosis, mild hyperplasia of the spinous layer, decreased pigment particles in the epidermal basal layer, and a small amount of lymphocyte infiltration in the superficial dermis and around the blood vessels. Vitiligo treatment was mainly preventing the immune system from damaging the melanocytes so that melanocytes could normally produce the melanin particles, and the number of melanin particles was increased so that the skin gradually returns to normal.

### 3.3. Changes in Blood Biochemical Indexes of Patients

Patients in the control group, group A, group B, and group C were treated by external application of calcipotriol ointment, that of MEBO, that of MEBO combined with blood transfusion, and the microneedle introduction of MEBO combined with blood transfusion, respectively. TP, ALB, and GLB were measured at the 1st, 3rd, 5th, and 7th weeks of treatment (Figure 4).  Figure 4(a) shows the changes in TP content of the four groups at different periods. There was no considerable difference in the TP content among the four groups after 1 and 3 weeks of treatment (*P* > 0.05). The TP content in groups B and C gradually increased with the extension of treatment time, and the increase rate was quite fast after the 3 weeks of treatment. The TP content of group C (62.3 ± 3.3 g/L and 64.3 ± 2.88 g/L) was observably higher than that of the control group (51.3 ± 3.17 g/L and 52.4 ± 3.17 g/L) and group A (52.6 ± 2.91 g/L and 51.8 ± 2.98 g/L) at the 5th and 7th weeks after treatment (*P* < 0.05). The TP content in group B at the 5th and 7th weeks was higher than that in the control group and group A, which was lower than that in group C (*P* < 0.05).

RETRACTED

Figure 4(b) show the changes in ALB content of the four groups at the different periods after treatment. The ALB content of patients in the four groups increased gradually with the extension of treatment time, and that in groups B and C increased fast. There was no significant difference in the content of patients in the first three weeks (*P* > 0.05). The ALB content in group C (42.9 ± 3.28 g/L and 45.3 ± 3.1 g/L) was signally higher than that in the control group (41.8 ± 3.44 g/L and 41.9 ± 3.23 g/L) and group A (41.3 ± 2.91 g/L and 42.1 ± 3.02 g/L) at the 5th and 7th weeks after treatment, and it was markedly higher than that in group B at the 5th week (*P* < 0.05).

Figure 4(c) shows the changes in GLB content of the four groups at the different periods after treatment. There was no substantial change in the GLB content of the four groups with the extension of treatment time. Furthermore, the differences were statistically insignificant in the GLB content of the four groups during the different periods after treatment (*P* > 0.05).

### 3.4. The Skin Improvement of Patients

Figure 5 shows the improvement of skin symptoms of patients in the control group, group A, group B, and Group C after treatment. The skin of patients with vitiligo had depigmentation spots, which were milky white and light pink, and the surface was smooth without rash. The white plaque's peripheral skin was darker than normal skin. One or more white plaques were linked into a piece after the white plaque was extended, resulting in a huge white plaque with an uneven shape. Multiple milky white patches, single patches the size of a nail cap, in a round or irregular shape, smooth surface, and no symptoms were the most prevalent vitiligo lesions. White plaques were usually found on the skin of the face, neck, back, upper limbs, and abdomen, all of which were easily exposed to light and were damaged. Figures 5(a)–5(d) show the skin manifestations of the affected parts of the four patients treated with different methods. In the control group, after three courses of external application of calcipotriol ointment, the patient's back plaque was not improved notably, and it was even slightly expanded. In group A, the area of white plaques was observably reduced after the external treatment of MEBO, and the color of the skin around plaques gradually returned to normal. After the external application of MEBO combined with blood transfusion, the area of white plaques in group B was also greatly reduced, with an obvious trend of improvement. Patients in group C were treated with microneedle injection of MEBO combined with blood transfusion, and the white plaques on the back were signally reduced or even disappeared, and the color of the skin around the plaques gradually returned to normal, which indicated that the treatment effect was good.

RETRACTED

### 3.5. Evaluation of Therapeutic Effect

The therapeutic effect was evaluated according to four grades, namely, cure, marked effectiveness, effectiveness, and ineffectiveness.  Figure 6 shows the number of patients in each group who were evaluated as the grades of cured, marked effectiveness, effectiveness, and ineffectiveness, and it also shows the comparison of cure rates among the four groups. The efficacy evaluation of patients in the control and group A was low, with no cured patients among them. There were two examples of marked effectiveness and five cases of effectiveness in the control group. Three patients in group A had substantial effectiveness, and three patients had efficacy, and the rest were ineffective. There were 2 cured patients in group B and 5 in group C. Besides, there were 3 cases of marked effectiveness and 3 cases of effectiveness, and only 1 patient in group C was assessed as ineffective treatment. The cure rates of groups C and B (93.33% and 66.67%) were higher than those of the control group and group A (40% and 46.67%), and group C was manifestly higher than group B (*P* < 0.05) (Figure 6(e)).

### 3.6. Comparison of Wound Healing Rate of Patients

The wound healing rate was calculated by measuring the area of skin plaques before and after treatment (Figure 7). With the prolongation of treatment time, the patient's wound area gradually decreased, so the wound healing rate increased. The increase of groups B and C was faster than that of the other two groups. The wound healing rates of group C at the 3rd, 5th, and 7th weeks after treatment (38.44%, 56.6%, and 90.23%) were higher than those of the control group, group A, and group B (*P* < 0.05). The wound healing rate of group B at the 5th and 7th weeks after treatment was higher than that of the control group and group A (40.3% and 75.8%) (*P* < 0.05).

## 4. Discussion

Vitiligo is characterized by depigmentation of the skin, which appears milky white or pale pink. The white patches will grow or enlarge as the disease progresses, eventually forming plaques [23]. Depigmentation plaques are common in vitiligo, and they have a smooth surface with no rash and a darker edge than normal skin. The patient's face, neck, arms, limbs, and back are easily exposed to light at the start of the disease, and the wounded skin appears in several small patches. Each spot gradually increases and connects to form a large white plaque with an irregular shape. It has a great impact and confusion on the image and psychology of patients [24, 25]. Histopathological examination is generally performed, that is, small pieces of suspicious lesions are removed and stained to observe their morphology under a microscope. Pathology is the study of disease, while histology is the study of tissues. The study of tissues connected to disease is known as histopathology. The tissue evaluated by the pathologist is described in a histopathology report. It can recognize the characteristics of cancer under a microscope. A biopsy report or a pathology report is other name for a histopathology report. Vitiligo can be diagnosed if the melanocytes and melanocyte granules decrease or even disappear under the microscope [26]. The major goal of this disease's treatment is to get the white plaques and skin back to normal. To prevent future damage to melanocytes, the immune system is disrupted (most commonly by external administration of glucocorticoid ointment or external immunosuppressant), and the melanocytes revert to normal and create melanin particles. An increase in the number of melanin particles can gradually restore the color of skin plaques to normal [27, 28]. Moreover, through the transplantation of melanocytes or normal cells, the extracted melanocytes are cultured and transplanted to the white plaque area for treatment [29]. In recent years, with the continuous improvement of the medical level, microneedle therapy has been gradually known and widely used in the medical field. Nofal et al. [30] found that the microneedle had the characteristics and advantages of precisely adjustable depth and real-time monitoring, and the depth and energy of the microneedle could be adjusted according to the different degrees by penetrating the skin with the microneedle. The tip of the microneedle penetrated the skin to introduce drugs, which not only improved the utilization value of drugs to achieve the effect of targeted therapy but also effectively avoided epidermal stimulation. Furthermore, the intelligent monitoring of the microneedle was helpful to prevent damage to the skin due to the excessive output energy that ensured the safety and reliability of the treatment process to a certain extent [31].

RETRACTED

Patients with anemia generally show that both the total protein and haemoglobin are lower than the normal value, and the haemoglobin content of patients with extremely severe anemia was lower than 30 g/L [32]. According to the treatment combined transfusion for anemia, TP and ALB levels in group C were remarkably higher than those in the control group and group A at the 5th and 7th weeks after treatment (*P* < 0.05). Blood transfusion therapy and transfusion nursing could improve the symptoms of patients with anemia to a certain extent. Furthermore, the MEBO, which helped to enhance the proliferation and differentiation of epidermal stem cells, was employed for the treatment of patients with severe anemia worsened by vitiligo under the medical technology hypothesis of skin regeneration in situ. The results reflected that the cure rates of group C and group B (93.33% and 66.67%) were higher than those of the control group and group A (40% and 46.67%), and group C was higher than group B (*P* < 0.05). The cure rate of patients with vitiligo treated with microneedle injection of MEBO was notably higher than that treated with MEBO externally. The wound healing rates of group C at the 3rd, 5th, and 7th weeks after treatment (38.44%, 56.6%, and 90.23%) were higher than those of the control group, group A, and group B (*P* < 0.05). The wound healing rate of group B at the 5th and 7th weeks after treatment was greatly higher than that of the control group and group A (40.3% and 75.8%) (*P* < 0.05). This was similar to the results of Birlea et al. [33]. As a result, MEBO promoted wound healing, ulcer healing, and anti-inflammation, as well as having a therapeutic effect on vitiligo. Because the microneedle could penetrate the skin through the activation of nerves, the therapeutic impact of drug therapy by microneedle in group C was considerably superior to that of external drug therapy. As a result, it had a therapeutic impact on the vitiligo-affected areas.

## 5. Conclusion

Patients with severe anemia exacerbated by vitiligo were chosen as study participants, and they were treated with MEBO external application combined with blood transfusion and MEBO microneedle injection combined with blood transfusion. The therapeutic efficacy of microneedle injection combined with blood transfusion in the treatment of severe anemia complicated by vitiligo was investigated by comparing the recovery of various blood indices and skin white plaque. The results reflected that microneedle injection combined with blood transfusion had a good therapeutic effect on patients with severe anemia complicated with vitiligo based on regenerative medical technology, which was helpful to improve the blood indexes and skin plaques of patients and had a good clinical adoption effect. Nonetheless, in this experiment, microneedle injection and blood transfusion are employed to treat patients with vitiligo and anemia, and the efficacy of a single disease is not evaluated for the treatment modalities, which may have an impact on the final evaluation indexes. This aspect needs to be optimized and improved in the subsequent explorations, and it will be further investigated.

RETRACTED

## Figures and Tables

**Figure 1:** Principle of the drug introduced by microneedles: (a) principle of the drug introduced by the microneedles; (b) skin melanocytes.

**Figure 2:** Blood indexes of patients before treatment: (a) the absolute values of white blood cells, neutrophils, and the total number of lymphocytes; (b) comparison of ALB among the four groups; (c) comparison of CLB among the four groups.

**Figure 3:** Microscopic images of the skin of patients with vitiligo: (a, b) images with magnification (×10); (c, d) images with magnification (×40); (e, f) images with magnification (×100).

**Figure 4:** Changes in patients' blood indexes after treatment: (a) changes in TP; (b) changes in ALB; (c) changes in GLB. Note: *a* meant that compared with the control group, *P* < 0.05; *b* meant that compared with group A, *P* < 0.05; *c* meant that compared with group B, *P* < 0.05.

**Figure 5:** Improvement of skin symptoms of patients: (a–d) the control group, group A, group B, and group C.

**Figure 6:** Evaluation of the therapeutic effect of patients in the four groups: (a–d) the control group, group A, group B, and group C; (e) comparison of the cure rate among the four groups. Note: *a* meant that compared with the control group, *P* < 0.05; *b* meant that compared with group A, *P* < 0.05; *c* meant that compared with group B, *P* < 0.05.

**Figure 7:** Comparison of wound healing rate of patients in the four groups. Note: *a* meant that compared with the control group, *P* < 0.05; *b* meant that compared with group A, *P* < 0.05; *c* meant that compared with group B, *P* < 0.05.

**Table 1:** Evaluation criteria for therapeutic effect.

Degree of cure	Symptoms
Cure (A)	The skin of the white plaques returned to normal without abnormal symptoms.
Marked effectiveness (B)	The white plaques were partially improved, and more than 50% of skin color was restored.
Effectiveness (C)	The skin was improved, and less than 50% of skin color returned to normal.
Ineffectiveness (D)	There were no obvious differences before and after treatment and no improvement in white plaques.

## Data Availability

The datasets used and/or analysed during the current study are available from the corresponding author upon request.
